RETRACTED

# Online Disease Identification and Diagnosis and Treatment Based on Machine Learning Technology

**DOI:** 10.1155/2022/6736249

**Published:** 2022-04-12

**Authors:** Feng Hao, Kai Zheng

**Affiliations:** Jilin Medical University, Jilin 132013, China

## Abstract

The article uses machine learning algorithms to extract disease symptom keyword vectors. At the same time, we used deep learning technology to design a disease symptom classification model. We apply this model to an online disease consultation recommendation system. The system integrates machine learning algorithms and knowledge graph technology to help patients conduct online consultations. The system analyses the misclassification data of different departments through high-frequency word analysis. The study found that the accuracy rate of our machine learning algorithm model to identify entities in electronic medical records reached 96.29%. This type of model can effectively screen out the most important pathogenic features.

## 1. Introduction

The background of this study was that the Internet medical service has a large amount of structured information such as diseases and hospitals, but the service to users is very limited. Most service sites only offer features such as online searches and consultation with doctors. Some websites offer simple self-diagnosis services. However, most only allow users to enter symptom keywords. The list of diseases given by the system is very long. Therefore, this paper proposes a method for extracting disease symptom keywords by a related machine learning algorithm. The application of this method can effectively retrieve information for intelligent recommendation of doctors and hospitals and greatly improve the efficiency of patients' medical treatment. It is of great significance and can effectively improve the medical environment of the hospital, but the disadvantage is that not every patient can use the system proficiently, and it needs a lot of operation training for the system later to be familiar with the use of the system.

The method adopted in this paper is that the system integrates machine learning algorithms and knowledge graph technology to help patients conduct online consultations. The power of this method is to effectively improve the level of urban medical care and services. The system analyses the misclassified data of different departments through high-frequency word analysis. In the later stage, the overall accuracy of this method is improved to more than 90%, which has a very significant effect [1].

To this end, this paper proposes a design and implementation method for constructing an inquiry recommendation system based on knowledge graphs, deep learning, and social media. We design the structured disease information of the web site for seeking medical advice to construct a “disease-symptom” knowledge map. We provide users with disease self-diagnosis services from various aspects of information. At the same time, the system uses the structured information of the knowledge graph to mine the potential diseases that the user may suffer from to enrich the recommendation options. We used the review data of the good doctor web site as a sample. We combined it with the existing service quality evaluation indicators to analyse the service quality of doctors in various hospitals in Beijing. We provide users with doctor and hospital recommendation services from multiple dimensions.

RETRACTED

## 2. Related Work

### 2.1. Disease Diagnosis Algorithm

Traditional disease diagnosis includes two types of methods based on algebraic operations and based on recommendation systems. It is generally accepted that many incomplete, uncertain, and inconsistent information in medical diagnosis. Therefore, many scholars use FS (fuzzy set) and NS (neutron sophist) to model the association between symptoms and diseases. At the same time, they compared the similarity between the FS or NS of the patient's symptoms and different diseases to diagnose the user's disease. With the popularity of machine learning, more and more scholars are trying to use machine learning technology to complete the task of disease diagnosis. Some scholars have used the back-propagation algorithm to train a single-layer neural network to complete the task of disease diagnosis based on patient symptom keywords and laboratory data. In addition, some scholars use medical images to identify possible diseases for patients. Some scholars use a convolutional neural network (CNN) to identify the occurrence of myocardial infarction. Some scholars also used CNN to complete the classification of skin cancer.

Comprehensive analysis of FS-based and NS-based disease diagnosis algorithms requires careful conditions modelling. This is far from the natural language text input by the user and is inconvenient for the user to use. The recommender system method requires many users' historical diagnosis and treatment data. This involves user privacy. Moreover, the above two methods do not consider the influence of age, gender, etc., on disease diagnosis.

### 2.2. Medical Knowledge Graph

A knowledge graph is a structured semantic knowledge base. This method describes concepts and their interrelationships in the physical world in symbolic form. Its basic unit is the “entity-relation-entity” triplet. It can also be an entity and its related attribute-value pairs, and the entities are interconnected through relationships to form a networked knowledge structure. The medical knowledge graph is a subset of the knowledge graph. Academia has carried out a lot of research on its construction methods and application scenarios. Specific medical service needs usually require the construction of a specific medical knowledge graph. At present, the technology of constructing knowledge graphs from EHR data is quite mature. These methods generally require the extraction of medical concepts from the semistructured text. The process involves natural language processing means such as machine learning. This method is more complicated. According to this paper's functional requirements of disease diagnosis, we only need to build a “disease-symptom” knowledge map. We can greatly reduce the complexity of building a knowledge graph by using many existing and reliable sources of structured disease information on the Internet.

RETRACTED

### 2.3. Analysis Technology Related to Medical Reviews

Sentiment analysis is the extraction and analysis of personal information such as people's opinions, emotions, and emotions about goods, services, organizations, people, events, and attributes. Sentiment analysis of medical reviews can be roughly divided into two categories: sentiment polarity analysis and sentiment attribute extraction.

Some scholars build a learning model on the comments of CSN (cancer survivors' network). They perform binary classification on the sentiment polarity of text to model the change of the user's emotional state and assist the community in providing better services. Some scholars combined the knowledge of the diabetes medical model and used N-gram to classify the sentiment polarity of diabetes-related tweets. Some scholars constructed a latent Dirichlet allocation (LDA) model based on the review data of the good doctor medical web site from 2006 to 2014. They extracted topic models such as curative effect and seeking medical treatment and conducted simple sentiment analysis.

Sentiment analysis techniques for comprehensive analysis of medical reviews are not advanced. None of them use the current popular deep learning model. Much of the work stops at analysing emotions themselves. They did not mine the available information further from the emotional information [2]. This paper will further mine emotional information combined with medical service evaluation indicators. We build an evaluation model for doctor-hospital service quality and use the evaluation model for recommendation services.

### 2.4. Design and Implementation of Consultation Recommendation System

The architecture diagram of the consultation recommendation system constructed in this paper is shown in Figure 1. The recommender system accepts symptom information input by the user. The content includes symptom keywords (required), symptom description, age, gender, etc. The final recommended results include three diseases and the corresponding recommended hospitals and doctors. The recommendation system mainly includes two services: disease diagnosis service and doctor recommendation service. The recommended steps consist of four steps in total. They are constructing disease candidates, expanding disease candidates, screening and sorting, and doctor-hospital recommendations. The implementation of the consultation recommendation system will be explained in turn.

RETRACTED

### 2.5. Building a Knowledge Graph

In this paper, the data from the website of seeking medical treatment and asking for medicine are selected as the source to construct a knowledge map. The web site seeking and seeking medicine is an Internet medical and health service platform. This article uses the information on 8802 diseases published on seeking medical advice. The content of this study mainly includes disease symptom description, disease symptom keywords, disease-susceptible population, disease incidence, disease department, disease complications, and other information.

Since most of the information on the web site for seeking medical treatment and seeking medicine is structured, a simple reprocessing is carried out in this paper. We mainly further extracted information such as the gender of the susceptible persons and the age of the susceptible persons from the susceptible population [3]. The age is based on the new age segment information of 360 Encyclopaedia and slightly modified. The aging stage is divided into 7 age groups: foetuses, infants, children, adolescents, youth, middle-aged, and elderly. Combined with the functional requirements of this paper, the knowledge graph structure finally designed in this paper is presented in Tables 1 and 2.

This paper uses the Neo4 graph database to store knowledge graphs. After the construction is completed, the knowledge graph contains 15,418 entities and 85,303 relationships.

### 2.6. Analysis of Medical Reviews

This article selects good doctor web site reviews as the data source. This article uses public data from the Good Doctor web site in 2018 and 2019. The content includes 133,667 reviews of online doctors in major hospitals.

This paper reprocesses the comment data of the Good Doctor web site to remove invalid Chinese and English characters. We use the Python third-party open-source library zhconv to convert the comment text to traditional and simplified. At the same time, we fixed some common mistakes in the colloquial expression of comment text. This article uses the Python third-party open-source library by corrector to correct the language error of the comment text.

RETRACTED

This paper starts from the SERVQUAL model to label the review data. This paper also fine tunes the SERVQUAL model and gives the principles of comment annotation. Since the Good Doctor web site data rarely involves comments on the evaluation of hospital hardware facilities and the clothing of medical staff, the Tangibles evaluation dimension is discarded. In addition, because the evaluation contents of responsiveness and empathy in the medical review data are too similar, this paper combines the two into one evaluation dimension. It records it as R&E [4]. Reliability corresponds to the description of efficacy in the review. Common expressions include “the condition has improved,” “the condition has worsened,” and so on. The R&E corresponds to the description of the doctor's medical attitude in the review. Common expressions include “the doctor is very patient and amiable,” “the doctor is very impatient,” etc. Assurance corresponds to the patient's overall assessment of the doctor's level of care in the review. Common expressions include “superior medical skills” and “average level.” There are three sentiment polarities annotated for each dimension: positive, neutral, and negative. A total of 6019 comments were marked.

This paper uses the BERT model for patient review analysis. We divide the annotation data set into training sets and validation set according to the ratio of 9 : 1. The final performance on the validation set is presented in Tables 3–5 [5]. The accuracy rates of the BERT model in the 3 dimensions are 78.4%, 88.1%, and 93.4%. The recall rates are 86.7%, 87.5%, and 97.2%, respectively. Since the third dimension lacks ground-truth negative review data, the absolute precision and recall calculations eliminate this part and work well.

## 3. Disease Diagnosis Services

### 3.1. Construction of Disease Candidates

This part mainly matches the diseases in the knowledge graph according to the keyword information input by the user. We rank possible diseases by disease incidence and keyword match. Keyword matching degree has higher priority in sorting. We screened the top 15 diseases as candidates [6].

### 3.2. Expanding Disease Candidates

This paper chooses to train the knowledge graph embedding with the Trans D model, to improve the accuracy of disease diagnosis. This model is developed on Trans E, Trans H, and Trans R. The Trans E model considers the relation vector *r* to be the translation of the head entity vector *h* to the tail entity vector *t*, namely, *h*+*r* ≈ *t*.

RETRACTED

Where *h* represents the head entity vector, *r* represents the relation vector, and *t* represents the tail entity vector. Because the model assumes that the same entity is represented under any relationship, the Trans E model performs well in dealing with one-to-one relationships. However, this model is slightly weak for complex relationships such as one-to-many and many-to-many. For this reason, the Trans H model believes that the head entity vector and the tail entity vector need to be projected on the hyperplane of the relation vector, namely:

(1) $$\begin{array}{c} h_{⊥}=h-\omega_{r}^{T}h\omega_{r};t_{⊥}=t-\omega_{r}^{T}t\omega_{r}. \end{array}$$

Then, set up:

(2) $$\begin{array}{c} h_{⊥}+r\approx t_{⊥}, \end{array}$$

where *ω*_*r*_ represents the normal vector of the hyperplane of relation vector *r*. The drawback of the Trans H model is that it still assumes that entities and relations are in the same semantic space. This limits its expressiveness. On this basis, the Trans R model further uses the projection matrix (*M*_*r*_) to complete the projection operation.

(3) $$\begin{array}{c} h_{⊥}=h-M_{r}h;t_{⊥}=-M_{r}t. \end{array}$$

The projection matrices given for the Trans R model for the same relation are the same. It does not take into account the differences between head and tail entities. Its projection operation involves matrix calculations, which greatly increases the training complexity. The Trans D model, on the other hand, considers projections to be interactions between entities and relationships. In addition, the computational complexity of Trans D is lower than that of Trans R. It gives the projection matrix and *h*_⊥_ and *t*_⊥_ are calculated as follows:

(4) $$\begin{array}{c} M_{r}^{1}=\omega_{r}\omega_{h}^{T}+I;M_{r}^{2}=\omega_{r}\omega_{t}^{T}+I,\\ h_{⊥}=h-M_{r}^{1}h;t_{⊥}=t-M_{r}^{2}h. \end{array}$$

This paper uses Open KE to implement the Trans D model to give the vector representation of relations and entities from the global graph structure information. We give the disease most similar to each disease in the candidate set according to the proximity of Euclidean distance. We add it to the candidate set [7]. The purpose is to mine potential diseases that users may suffer from and enrich recommendation options. This improves the accuracy of disease diagnosis.

### 3.3. Filter Sort

This section scores and ranks the diseases in the candidate set according to the 4 dimensions entered by user *i*. We select the top 3 diseases to recommend to users. The scoring formula for a disease *j* is:

(5) $$\begin{array}{c} S_{j}=S_{\text{age}}+S_{\text{sex}}+S_{\text{key}}+S_{\text{des}}. \end{array}$$

Among them, *S*_age_, *S*_sex_, *S*_key_, *S*_des_ represent the similarity between disease *j* and user *i* input in terms of age of susceptible population, gender of susceptible population, symptom keywords, and disease description, respectively. The age and gender similarity judgments are based on simple string matching. The formula for calculating *S*_key_ is as follows:

(6) $$\begin{array}{c} S_{\text{key}}=\frac{\left|{\text{Key}}_{i}\cap {\text{Key}}_{j}\right|}{\left|{\text{Key}}_{i}\right|}. \end{array}$$

Key_*i*_, Key_*j*_ represent the symptom keyword set input by user *i* and the symptom keyword set owned by disease *i*, respectively [8]. *S*_des_ is calculated by the disease candidate set. Its description is as text collection D. We tokenize it and remove Chinese stop words. We assume that the final vocabulary set is {*t*_1_, *t*_2_,…, *t*_*n*_}, and then, calculate the TF-IDF values of all words according to the TF-IDF algorithm for each text in the text set to obtain the TF-IDF matrix:

(7) $$\begin{array}{c} M=\left[\begin{array}{cccc} tfi\;df_{11} & tfi\;df_{21} & \cdots & tfi\;df_{n1}\\ tfi\;df_{12} & tfi\;df_{22} & \cdots & tfi\;df_{n2}\\ \vdots & \vdots & \vdots \\ tfi\;df_{1|D|} & tfi\;df_{2|D|} & \cdots & tfi\;df_{n|D|} \end{array}\right]. \end{array}$$

*tfi*  *df*_*ij*_ represents the TF-IDF value of word *t*_*i*_ in a text *D*_*j*_. Finally, the TF-IDF vector of the disease symptom description input by the user is also calculated by a similar method. Then, the row vector in the matrix *M* obtains the *S*_des_ of each disease in the candidate set according to the cosine similarity calculation method.

RETRACTED

### 3.4. Doctor Referral Service

This paper has performed sentiment polarity analysis on reviews using the BERT model. We got the number of positive, negative, and neutral reviews for 3 dimensions in all doctor reviews. This paper gives the scores of doctors and even the corresponding departments based on the Wilson interval method. Wilson's formula is as follows:

(8) $$\begin{array}{c} \text{Score}=\frac{p+\left(z_{a}^{2}/2n\right)-\left(z_{a}/2n\right)\sqrt{4n\left(1-p\right)p+z_{a}^{2}}}{1+\left(z_{a}^{2}/2n\right)}. \end{array}$$

*p* is the positive rating, *n* is the total number of reviews, and *z*_*a*_ is the quantile. It is used to express the confidence of this score. Wilson's interval method has a good degree of discrimination and also has the following properties:

1. Score normalization.
2. When *p* is constant, the larger *n* is, the decreasing speed of the numerator is less than the decreasing speed of the denominator. The higher the score at this time, the score approaches *p* as *n* approaches infinity. In other words, the rating method will consider the positive rating to be reliable when the total number of reviews is high. In addition, when the total number of reviews is low, the positive rating is considered unreliable.

RETRACTED

This paper chooses *z*_*a*_ to be 2 (that is, the confidence level is about 95%) and makes a slight modification to the Wilson interval method. The premise of the Wilson interval method is that there are only positive and negative comments, but there are neutral comments in the actual application scenario of this article. Therefore, this paper regards half of the neutral reviews as positive when calculating the favourable rate. The other half are classified as negative reviews. After obtaining the scoring information of doctors and hospital departments, we select the corresponding department according to the disease information. At this time, the system recommends the 4 best hospitals. Each hospital recommends the 4 best doctors.

## 4. Verification

### 4.1. Validation of the Disease Diagnosis Algorithm

This article comprehensively presents the possible diseases from the four perspectives of age, gender, keywords, and symptom description. At the same time, this paper uses the structural information of the knowledge graph to give the potential diseases that the user may suffer from. This enriches the recommendation options. At present, there is no similar work in industry and academia. Therefore, this paper adopts the practice of constructing a test set to verify the accuracy of the disease diagnosis algorithm [9].

This article selects 50 common diseases in various departments from the web site of seeking medicine and asking for medicine, such as colds, rhinitis, and otitis media. Then, combined with the disease symptom information on the Baidu Baike web site, it was reorganized using natural language. We input it as a hypothetical user symptom description. Combined with the keyword information of the web site for seeking medical advice, we construct user test cases. This is the test set *T*_1_. The test set *T*_2_ is obtained by adding a certain amount of complication keyword information for each disease in the test set *T*_1_ as confusion. Complication information is obtained from the Seek for Medicine web site.

The results of running the algorithm on the test set are presented in Table 6. After adding the complication information, the algorithm's accuracy has dropped significantly. On the one hand, it is because of the interference of extra information. On the other hand, some diseases do not have many keywords due to their symptoms. The addition of the complication keyword amplifies the confounding effect. In addition, due to the different sources of disease information on Baidu Baike and the web site for seeking medical treatment and medicine, the descriptions of the same disease are not the same. For example, Baidu Encyclopaedia gives a variety of classifications for the disease cheilitis, such as granulomatous cheilitis and actinic cheilitis. The web site of seeking medical advice only gives general symptom descriptions for cheilitis. This is also one of the reasons why the accuracy rate is not ideal. Although the algorithm cannot accurately diagnose the patient's disease in some cases, the recommended results include similar diseases or diseases in the same department [10].

RETRACTED

### 4.2. Validation of Doctor Recommendation Algorithms

The verification of this part takes the form of a questionnaire. The questionnaire is mainly for Peking University students [11]. The questionnaire selected 3 kinds of diseases, such as respiratory infection, urticaria, and rhinitis, relatively common among students. Each disease sets the same questions. Ask the subject if they have had the disease whether the disease has been treated in the Beijing area. Students recognize the doctor and hospital recommendations given by the recommendation system in this article. Finally, 57 questionnaires were recovered. The verification results are presented in Table 7.

Among all the survey subjects who had suffered from the disease and visited the Beijing area, there was only 1 case of rhinitis in the wrong doctor recommendation. There were only 2 cases of hospital recommendation errors and 3 cases of doctor recommendation errors in the urticaria part [12]. There was only 1 case of hospital recommendation error in the respiratory tract infection part and 1 case of doctor recommendation error. Comprehensive questionnaire results the accuracy of the consultation recommendation system proposed in this paper for hospital recommendations is 93.57% [13]. The system recommends doctors with an accuracy of 90.91%. The application of the system works well.

## 5. Conclusion

This paper designs and implements a medical consultation recommendation system. In this paper, a “disease-symptom” knowledge map is constructed to provide users with disease self-diagnosis services. At the same time, we use the deep learning model to give the hospital doctor's service quality evaluation model to provide users with better recommendation services. The system constructed in this paper allows users to input various information such as gender. In this way, a reasonable disease recommendation can be comprehensively given. This paper leverages the structured information of knowledge graphs. The model can mine potential diseases that users may have and enrich recommendation options. This paper also innovatively links medical reviews and medical service quality. This provides users with a more open and reasonable recommendation service.

RETRACTED

## Figures and Tables

**Figure 1:** Framework diagram of consultation recommendation system.

**Table 1:** Knowledge graph entities.

Entity	Attributes
Disease	Disease description, the incidence
Symptom keyword	None
Department	None
Age	None
Gender	None

**Table 2:** Knowledge graph relationships.

Relation	Head entity	Tail entity
Have symptoms	Disease	Symptom's keyword
Have complications	Disease	Disease
Department	Disease	Department
Susceptible age	Disease	Age
Predisposing gender	Disease	Gender

**Table 3:** Reliability dimension verification results.

Emotional polarity	Positive (prediction)	Neutral (predicted)	Negative (prediction)
Positive (real)	76	12	3
Neutral (true)	15	344	59
Negative (true)	1	6	84

**Table 4:** R&E dimension validation results.

Emotional polarity	Positive (prediction)	Neutral (predicted)	Negative (prediction)
Positive (real)	233	17	3
Neutral (true)	25	199	18
Negative (true)	3	3	179

**Table 5:** Assurance dimension validation results.

Emotional polarity	Positive (prediction)	Neutral (predicted)	Negative (prediction)
Positive (real)	148	3	0
Neutral (true)	16	421	0
Negative (true)	0	12	0

**Table 6:** Validation accuracy % of disease diagnosis algorithm.

Validation metrics	T1 test set	T2 test set	Average accuracy
Hit@3	80	68	74
Hit@5	88	74	81
Hit@10	94	80	87

**Table 7:** Questionnaire survey results.

Validation metrics	Respiratory infection	Hives	Rhinitis
Hospital recommendation error	7	1	3
Doctor recommends correct	54	61	65
Select the total number of doctors	61	68	69
Number of people who have had the disease	18	20	28
Number of people who have been treated for the disease in Beijing	11	15	18

## Data Availability

The data used to support the findings of this study are available from the corresponding author upon request.
